The article "Vestibular Autorotation Test: The Differences in Peripheral and Central Acute Vestibular Syndrome" was retracted in 2023. Reasons: unreliable results or conclusions; lack of ethics approval or compliance; concerns about the data; concerns about the peer review.

# Vestibular Autorotation Test: The Differences in Peripheral and Central Acute Vestibular Syndrome

**DOI:** 10.1155/2022/8180013

**Published:** 2022-08-13

**Authors:** Nan Guo, Lijing Zhou, Yu Zhang, Xiuyu Fan

**Affiliations:** Electrophysiology Office, The Third Affiliated Hospital of Qiqihar Medical College, Qiqihar, China

## Abstract

**Objective:**

To evaluate the difference between the vestibular autorotation test (VAT) in the peripheral and central acute vestibular syndrome (AVS). *Methodology.* Patients with AVS diagnosed by clinical manifestation admitted to the third affiliated hospital of Qiqihar Medical College from January 2019 to January 2021 were enrolled and divided into peripheral AVS (peripheral group) and central AVS (central group) according to the results of the MRI examination.

**Results:**

A total of 332 patients with AVS were recruited, including 282 patients in the peripheral group and 50 patients in the central group. The horizontal gain of both groups showed a downward trend at 2–6 Hz. There was no significant change in the horizontal phase between the two groups at 2–6 Hz. The horizontal gain of the two groups was stable at 2–6 Hz with no significant changes in the horizontal phase between 2–6 Hz in both groups. The central group showed a significantly lower proportion of gain increase coupled with loss and a strikingly higher proportion of gain increase without a loss than in the peripheral group (all *P* < 0.001).

**Conclusion:**

The increased horizontal and vertical gain of VAT in patients with AVS is of high value in the diagnosis of ACS. Significant differences in the results of VAT in patients with central and peripheral AVS could provide a reference for diagnosis.

## 1. Introduction

Acute vestibular syndrome (AVS) features a host of clinical syndromes, including acute onset, long-lasting vertigo/dizziness, and progressive vestibular system dysfunction, with a single-phase duration [1, 2]. There is no application of Chinese medicine in AVS, but the application of Chinese medicine in vertigo is very popular. In the theory of Traditional Chinese medicine, vestibular migraine vertigo is classified as “headache,” “headwind,” and “vertigo” [2]. It is thought that it is mostly due to phlegm, wind, silt, and fire disturbance to clear the body, plus the body qi deficiency and kidney essence deficiency resulting in loss of nutrition of the marrow sea [3].

Clinically, the acute vestibular syndrome can be divided into peripheral and central vascular according to different etiologies. The peripheral acute vestibular syndrome includes vestibular neuritis, migraine, and Meniere's disease. Central vascular acute vestibular syndrome is mainly caused by cerebral ischemia. At present, the clinical diagnosis of central vascular acute vestibular syndrome mainly depends on the imaging data and clinical symptoms of patients, which challenge the diagnosis due to the complicated operation.

Although AVS is normally induced by vascular peripheral disease, acute vertigo caused by stroke requires great attention for its severe consequences [4]. The vestibule interacts with other systems of the body through reflex pathways to maintain coordination, among which the most important is the vestibulo-ocular reflex (VOR) [5]. The VOR pathway, as a key part of the vestibular function test, maintains visual clarity by regulating eye movement during head movement. The traditional modalities such as rotation tests and cold/heat experiments are limited to vestibular function at 0.0125–0.1 Hz, which is far below the daily activities frequency (2–5 Hz), and thus has poor diagnostic efficacy for vestibular function [6]. Vestibular Autorotation Test (VAT), as a method for vestibulo-ocular reflex, can detect vestibular function at 2–6 Hz. It has been widely used for the diagnosis of peripheral vestibular lesions but is rarely applied in acute vestibular syndrome [7, 8].

By studying the value of VAT in the diagnosis of AVS and analyzing it, this paper aims to provide an effective diagnostic method for AVS, and then provide a reference for the formulation of clinical treatment plans, and further improve the prognosis of patients.

## 2. Information and Methodology

### 2.1. General Information

Patients with the acute vestibular syndrome who were admitted to this hospital from January 2019 to January 2021 were selected as the study group, and 50 healthy patients who were matched in age and gender during the same period were selected as the control group. The healthy population is arranged into the control group, and the AVS patients are arranged into the study group. In addition, the AVS patients (study group) are divided into peripheral AVS (peripheral group) and central AVS (central group). Inclusion criteria were as follows: (1) 18–80 years old; (2) acute onset, vertigo/dizziness lasting for more than 24 hours; (3) first episode, and no symptoms such as dysphagia, cough in diet, and ataxia; (4) the patients and their families signed the informed consent form. Exclusion criteria were as follows: (1) recurrent vertigo syndromes such as benign paroxysmal positional vertigo and Meniere's disease; (2) consciousness disorder or concomitant mental disease that prevents cooperation with the examination; (3) with hearing impairment and refractive error; (4) with new evident symptoms of neurological deficits; (5) with MRI contraindications or refusal to MRI examination.

### 2.2. AVS Diagnosis

All patients underwent cranial MRI upon admission, and cranial MRI could be repeated after 72 hours if a central vestibular lesion was suspected. Etiologies were classified based on MRI findings and clinical manifestations. Peripheral AVS includes vestibular neuritis, migraine, and Meniere's disease, and central vascular VAS mainly includes cerebral ischemia. The etiology was determined based on their respective diagnostic methods [9–11].

### 2.3. VAT Detection

All subjects were tested by a vestibular autorotation meter (WSR, the US). The meter includes a control center, a signal receiver, and a head sensor. Patients' head and eye movements were recorded and analyzed by computer software, represented by mean and standard deviation. VAT data included head and eye movement at 2–6 Hz, and the results included gain (horizontal and vertical), phase (horizontal and vertical), and asymmetry. VAT was averaged three times in the horizontal and vertical directions at an interval of 18 s. The low-frequency data were used for calibration in the first 6 s, and the data were recorded to calculate the parameters in the late 12 s. Under normal conditions, the gain is close to 1. The reaction gain increases when the gain is greater than 1 and decreases when the gain is less than 1. Phase refers to the phase-time relationship between output and input, i.e. the speed of eyeball movement lagging behind the head movement, with a normal phase of 180°, 0–180° for phase lag, and 180–360° for phase overrun. Asymmetry represents the symmetry between bilateral eye movements, with a normal value of 10%. Over 10% means lesions were on the right side, and below 10% means lesions were on the left side [12]. In VAT detection, an increase in gain without concomitant decrease is a central AVS, and an increase in gain with concomitant decrease is a peripheral AVS.

### 2.4. Statistical Methods

SPSS 22.0 was used for data collation and statistical analyses, and GraphPad Prism 7.0 software was adopted for image rendering. Measurement data were expressed as mean standard deviation. Two independent samples *t*-test was used for intergroup comparison, and one-way analysis of variance and back testing was used for comparison at different times within the group. Enumeration data were expressed as rates, and the presence of statistical differences between groups was compared using the Chi-square test or Fisher's exact test. The difference was considered statistically significant at the threshold of *α* = 0.05.

## 3. Results

### 3.1. Baseline Data

As shown in Table 1, a total of 332 AVS patients were included in this study. The differences in the baseline data such as gender, age, underlying diseases, and bad habits between the two groups were not statistically significant (all *P* > 0.05).

### 3.2. VAT Gains at Different Frequencies

As shown in Figure 1, both groups presented declining horizontal gains at 2–6 Hz, and the peripheral group showed higher horizontal gains than the central group at 2 Hz, 3 Hz, 4 Hz, and 5 Hz (all *P* < 0.001). At 6 Hz, there was no significant difference in horizontal gains (*P* > 0.05).

### 3.3. VAT Horizontal Phase at Different Frequencies

As shown in Figure 2, there was no significant change in the horizontal phase between the two groups at 2–6 Hz, and the peripheral group was drastically lower than the central group in the horizontal phase at 5 Hz and 6 Hz (all *P* < 0.05). There was no significant difference in horizontal gains between the two groups at 2 Hz, 3 Hz, and 4 Hz (all *P* < 0.05).

### 3.4. VAT Vertical Gains at Different Frequencies

As shown in Figure 3, the horizontal gains of the two groups nearly leveled at 2–6 Hz, and the peripheral group showed markedly higher vertical gains than the central group at each frequency (all *P* < 0.001).

### 3.5. VAT Vertical Phase with Different Frequencies

As can be seen in Figure 4, there was no significant difference between the two groups of horizontal phases at 2–6 Hz, and the group peripheral group presented a dramatically lower vertical phase than the central group at 6 Hz (*P* < 0.001). The two groups showed a similar vertical phase at 2 Hz, 3 Hz, 4 Hz, and 5 Hz, respectively (*P* > 0.05).

### 3.6. VAT Experimental Results

As shown in Table 2, the peripheral group had a higher proportion of patients with increased gain accompanied by decreased gain and those without increased gain than the central group (all *P* < 0.001). There was no significant difference in phase delay or asymmetry between the two groups (all *P* > 0.05).

## 4. Discussion

AVS is a common neurological disease with a high prevalence. Among the “vertigo/dizziness” patients in the emergency department, AVS accounts for 10–20% with an incidence as high as 20% in the elderly over 60 years [13]. AVS has various etiologies, which are closely related to the destruction or stimulation of peripheral or central vestibular structures such as the labyrinth of the inner ear, vestibular nerve, cerebellum, vestibular nucleus, and the ascending region from the thalamus to the cerebral cortex. Peripheral AVS is more common in clinical scenarios [14], including Meniere's disease, vestibular neuritis, and otolith, and central AVS is characterized by cumulative ischemic strokes in the brain stem and cerebellum [15,16]. The proportion of peripheral AVS was significantly higher than that of central AVS in the present study, which was consistent with the results in previous studies.

The results of the present study showed a significantly higher horizontal gain of peripheral AVS patients than central AVS patients at the frequency of 2–6 Hz. The peripheral group presented a much lower horizontal phase than the central group at 5 Hz and 6 Hz, substantially elevated horizontal gains at the frequency of 2–6 Hz, and a dramatically lower vertical phase at 6 Hz. The clinical symptoms of the central vascular acute vestibular syndrome are complex, and it is difficult to distinguish it from peripheral acute vestibular syndrome by the clinical symptoms and imaging examinations alone. VAT is a method widely used in clinical practice to judge the vestibular function of patients which can detect the patient's small shaking head and nodding movements in a short time, and then test the vestibular eye movement reflex of the body including the cerebellum and visual function. VAT is painless, accurate, and fast, and is more complete than traditional low-frequency vestibular function testing. VAT is a novel test method for a vestibular function that evaluates the vestibular function and the oculomotor system function from five aspects, i.e., horizontal or vertical phase, horizontal or vertical gain, and asymmetry. VAT has been widely used in the diagnosis of AVS given its advantages of painlessness, high accuracy, time-efficient, and more comprehensive coverage compared with traditional low-frequency methods [17]. In the present study, there are significant differences in horizontal gain and vertical gain between peripheral and central AVS patients. The proportion of AVS patients with increased gain accompanied by decreased gain was significantly higher than those without an increased gain, demonstrating its value in the diagnosis of AVS. Central AVS, especially isolated posterior circulation stroke induced by AVS, requires timely treatment, however, it is difficult to be identified due to similar symptoms with peripheral AVS [18]. VAT contributes to distinguishing peripheral AVS from central AVS. Here, the central group saw a much lower proportion of increased gain accompanied by loss than the peripheral group, and a significantly higher proportion of increased gain without accompanied decrease. The reason may be attributed to the vestibular hyperreflexia caused by the weakening ability of central AVS to the inhibition of the cerebellum which serves as the second regulation center of vestibular-oculomotor reflex inhibiting the regulation of the extraocular muscle nucleus and vestibular nucleus. The three possible anatomical sites involved in central vascular AVS are as follows: the cerebellar nodules, the site where the eighth cranial nerve enters the brainstem at the pontomedullary symphysis, and the vestibular nucleus. These structures all receive vestibular afferents from the inner ear, so theoretically, a small infarct confined to these areas could cause vertigo without other neurological symptoms or signs. The vestibulo-ocular reflex belongs to one of the neural reflex systems. The cerebellar follicular lobe can detect the vestibular and extraocular muscles of the inner ear, and at the same time effectively regulate the error of the vestibulo-ocular reflex. And the second-order regulatory center of vestibulo-ocular reflex is the cerebellum, and its role is mainly to inhibit the regulation of the extraocular muscle nucleus and the vestibular nucleus. The central vascular acute vestibular syndrome will have a certain impact on the structure or function of the cerebellum of patients, and then weaken the inhibition of the cerebellum, which further promotes the hyperactivity of the vestibular eye movement reflex. In the present study, the detection rates of central AVS and peripheral AVS by VAT were 8 4.21% and 72.44%, respectively, which were at a relatively low level. The reason might be that elderly people are often complicated with chronic diseases such as hypertension and hyperlipidemia, which led to blood supply disorders such as internal auditory artery and thus abnormal VAT results [19, 20].

This study also has the following limitations. This study was a single-center study, and the investigators were not blinded, resulting in certain results bias. In addition, this study only compared the differences in VAT results between peripheral and central AVS, and did not compare the diagnostic value of the corresponding indicators of VAT.

In conclusion, the increased horizontal and vertical gains of VAT in patients with AVS are of high value in the diagnosis of acute vestibular syndromes. Significant differences in VAT results between central AVS patients and peripheral AVS patients could provide a reference for diagnosis.

## Figures and Tables

**Figure 1:** Comparison of VAT gains at different frequencies in two groups, ^*∗∗∗*^ represents *P*  <  0.001.

**Figure 2:** Comparison of VAT horizontal phase at different frequencies in two groups, ^*∗*^ stands for *P*  <  0.05, ^*∗∗∗*^ stands for *P* < 0.001.

**Figure 3:** Comparison of VAT vertical gains at different frequencies in two groups, ^*∗∗∗*^ represents *P*  <  0.001.

**Figure 4:** Comparison of VAT vertical phase at different frequencies in two groups, ^*∗∗∗*^ represents *P*  <  0.001.

**Table 1:** Comparison of general information between the two groups.

	Control group (*n* = 50)	Study group (*n* = 282)	*t*/*χ*2	*P*
Age	58.34 ± 12.34	60.26 ± 14.58	0.877	0.381
Gender (male/female)	32/18	192/90	0.323	0.570
Hypertension (yes/no)	22/28	158/124	2.475	0.116
Diabetes (yes/no)	20/30	136/146	1.154	0.283
Hyperlipidemia (yes/no)	19/31	128/154	0.940	0.332
Ischemic heart disease (yes/no)	8/42	30/252	1.205	0.272
Smoking (yes/no)	14/36	88/194	0.205	0.651
Alcohol (yes/no)	12/38	79/203	0.344	0.558

**Table 2:** Comparison of VAT experimental results between the two groups.

	Increased gain with a decrease	Increased gain without a decrease	Phase delay	Asymmetry
Peripheral group (*n* = 282)	0	4 (8.00)	12 (24.00)	16 (32.00)
Central group (*n* = 50)	190 (67.38)	152 (53.90)	48 (17.02)	87 (30.85)
*χ*2	—	39.52	1.397	0.026
*P*	<0.001^*∗*^	<0.001	0.237	0.871

*Note.* ^*∗*^ stands for Fisher precision test.

**Table 3:** VAT comparison between central and peripheral AVS patients.

	Increased gain with a decrease	Increased gain without a decrease	Phase delay	Asymmetry
Peripheral group (*n* = 282)	163 (72.44)	104 (46.22)	39 (14.72)	66 (29.33)
Central group (*n* = 50)	27 (47.37)	48 (84.21)	9 (15.79)	21 (36.84)
*χ*2	13.01	26.41	0.043	1.202
*P*	<0.001	<0.001	0.837	0.273

## Data Availability

The datasets used during the present study are available from the corresponding author upon reasonable request.
